# Teaching Quality Evaluation of Animal Science Specialty Based on IPSO-BP Neural Network Model

**DOI:** 10.1155/2022/3138885

**Published:** 2022-09-23

**Authors:** Liyan Chen, Lihua Wang, Chunyou Zhang

**Affiliations:** College of Animal Science and Technology, Inner Mongolia Minzu University, Tongliao 028000, China

## Abstract

Teaching quality evaluation is one of the most commonly used educational evaluation methods, which is used to evaluate teachers' teaching ability and teaching effect. In order to improve the effectiveness and accuracy of teaching quality evaluation, a BP neural network model based on improved particle swarm optimization (IPSO) is proposed. Firstly, the evaluation index system of teaching quality is constructed with teaching attitude, teaching content, teaching method, and teaching effect as indicators. Then, IPSO algorithm is used to optimize the weight and threshold of neural network to improve the performance of BP algorithm. Secondly, IPSO-BP algorithm is used for sample training to optimize the model structure. Finally, the model is used to evaluate the teaching quality of animal science-related courses in Inner Mongolia University for Nationalities. The results show that compared with the ordinary BP neural network model, the IPSO-BP model has fast convergence speed, good robustness, and strong global search ability, and the evaluation accuracy rate is 96.7%. It is feasible in the evaluation of teaching quality.

## 1. Introduction

Teaching quality is not only the lifeline of the survival and development of higher education but also an important link to measure the teaching management and teaching effectiveness of colleges and universities. Through the quantitative evaluation of teachers' teaching activities by different subjects, we can judge the teaching effect, test whether the expected teaching objectives have been achieved, and test the students' ability to accept the teaching process [1]. Teaching quality evaluation is a fuzzy nonlinear problem, which has the characteristics of wide evaluation content and many evaluation indexes. Therefore, there are often some problems in the evaluation process, such as imperfect evaluation index system, unscientific evaluation methods, and so on. Therefore, how to improve the scientificity and effectiveness of teaching quality evaluation is the focus of researchers.

Foreign scholars have studied the evaluation of teaching quality earlier. Among them, the teaching effect evaluation index system proposed by scholars Zhou is the most representative [2]. Later, scholars made continuous improvement on the evaluation methods. Fuzzy comprehensive evaluation method [3], grey system theory [4], analytic hierarchy process, and support vector machine are widely used to further improve the reliability of evaluation. Although these methods consider the corresponding relationship between teaching quality and evaluation indexes [5, 6], it is difficult to eliminate the problems of subjectivity and randomness in the process of evaluation, and they have some limitations on the nonlinear evaluation of teaching quality. Therefore, it is necessary to establish a scientific teaching quality evaluation index system according to the characteristics of different courses and students, measure the factors affecting teaching quality from multiple levels, angles, and directions, and establish an evaluation model based on intelligent control algorithm, so as to improve the accuracy of teaching quality and provide a scientific basis for teaching management and decision making.

BP neural network can simulate the nervous system of human brain, can accurately approximate any nonlinear function, has strong data analysis ability and self-learning ability, and is widely used in various fields [7]. In recent years, many scholars have been trying to apply it to the process of teaching quality evaluation, which has greatly improved the accuracy of teaching quality evaluation. However, because the descent learning method adopted by BP neural network is a local search method, the convergence speed is slow, which makes the neural network easy to fall into local minimum and have weak generalization ability.

Based on the existing research, this paper constructs an IPSO-BP neural network model, which uses particle swarm optimization algorithm to optimize the weight and threshold of neural network, so as to improve the performance of BP algorithm, shorten the training time of neural network, and improve the search efficiency and accuracy. At the same time, the trained IPSO-BP neural network model is used to evaluate the teaching quality of colleges and universities, verify the reliability and feasibility of the model, and provide a theoretical basis for examining teachers' teaching effect, improving teaching methods, and optimizing teaching management process.

## 2. Construction of Teaching Quality Evaluation Index System

### 2.1. The Role of Teaching Evaluation

#### 2.1.1. Teaching Effect Test

Teaching evaluation itself is also a kind of teaching activity, which can quantitatively evaluate teachers' teaching activities through different subjects, so as to determine the teaching effect, test whether teachers can complete the corresponding teaching tasks and achieve the expected teaching objectives, and test students' acceptance of the teaching process.

#### 2.1.2. Teaching Feedback and Guidance

Through the feedback of teaching evaluation information, teachers can understand their own teaching effect and students' learning situation, timely optimize the teaching mode, and modify the teaching means, so as to continuously improve the teaching quality and the effectiveness of classroom learning.

#### 2.1.3. Regulating Teaching Management

Teaching evaluation can be used to verify whether the school teaching management is standardized, institutionalized, and scientific, monitor teachers' teaching quality, and master students' learning dynamics, so as to adjust teaching plans and educational objectives and to improve the teaching quality evaluation system.

### 2.2. Teaching Quality Evaluation Index System

Because there are some individual differences between teaching participants and evaluators, it is difficult to draw scientific and effective conclusions by direct teaching evaluation. Therefore, it is necessary to establish a teaching quality evaluation system, find out the index factors that can directly reflect the teaching effect, and then establish an evaluation model based on the index factors, so as to carry out comprehensive evaluation [8].

Scientific and effective evaluation results depend on a reasonable and standardized index system. This paper establishes the evaluation index system of teaching quality through in-depth investigation. It includes four primary indicators: teaching attitude, teaching content, teaching method, and teaching effect, which are expressed by *A*_1_, *A*_2_, *A*_3_, and *A*_4_, respectively. It is subdivided into 16 secondary indicators, represented by *A*_11_, *A*_12_, *A*_13_,..., *A*_43_, and *A*_44_, respectively. At the same time, the index weight is allocated according to the expert experience and the actual teaching situation of the unit, as shown in Table 1.

## 3. BP Neural Network Model

### 3.1. Structure and Principle of BP Neural Network

Backpropagation (BP) is a multilayer feedforward network trained according to the error backpropagation algorithm. It can simulate the human brain nervous system and learn and modify the input information, so as to achieve objective and fair information output. Its model structure mainly includes input layer, hidden layer, and output layer. BP neural network continuously optimizes the network by modifying the thresholds between the input layer, hidden layer and output layer, so as to minimize the error between the output value and the target value. It is widely used in machine learning, artificial intelligence, information prediction and other fields [9].

BP neural network can approach any nonlinear function infinitely. Its learning process is divided into two stages: signal forward propagation and error backpropagation. When the signal propagates forward, the input sample is transmitted from the input layer, processed by the hidden layer, and then transmitted to the output layer. Compare the actual output results with the target output results. If they are inconsistent, it will turn to the backpropagation stage of error. Backpropagation is to transfer the output error back to the input layer in some form through the hidden layer, distribute the error to each neuron, and constantly correct the connection weight and threshold between each layer, so that the error decreases along the gradient direction until the output error reaches the preset accuracy or reaches the set maximum learning times [10]. BP neural network usually adopts three-layer network structure, as shown in Figure 1.

Let the input data and output data of training samples be *x*(*t*) and *y*(*t*), respectively, the input vector of BP neural network be *X*=(*x*_1_, *x*_2_, ⋯,*x*_*i*_)^*T*^, and *i* be the number of nodes in the input layer. The output vector of the output layer is *Y*=(*y*_1_, *y*_2_, ⋯,*y*_*k*_)^*T*^, and *k* is the number of nodes of the output layer.

The output expression of the hidden layer is

(1) $$\begin{array}{c} H_{j}=\overset{m}{\underset{i=1}{\sum }}\omega_{ij}x_{i}-\theta_{j}\text{.} \end{array}$$

Select the sigmoid function to build the mapping relationship, and the function expression is

(2) $$\begin{array}{c} f\left(x\right)=\frac{1}{1+e^{-x}}\text{,} \end{array}$$

where *ω*_*ij*_ is the weight between the input layer and the hidden layer; θ*j* is the threshold of the hidden layer; and *m* is the number of nodes in the hidden layer.

The output expression of the output layer is

(3) $$\begin{array}{c} L_{k}=\overset{k}{\underset{j=1}{\sum }}\omega_{jk}b_{j}-\theta_{k}\text{,} \end{array}$$

where *ω*_*jk*_ is the weight between the hidden layer and the output layer and *θ*_*k*_ is the threshold of the output layer.

Define the error between the actual output and the target output as

(4) $$\begin{array}{c} E=\overset{m}{\underset{k=1}{\sum }}{\left(L_{k}-Z_{k}\right)}^{2}\text{,} \end{array}$$

where *L*_*k*_ is the actual output and *Z*_*k*_ is the target output.

The learning and training process of BP neural network is the process of continuously adjusting the weight and threshold according to the error *E*, so that the actual output of training gradually converges to the expected output until the iteration reaches the set upper limit or the prediction accuracy reaches the threshold.

The gradient descent method is applied to update the weight, and the expression is [11]

(5) $$\begin{array}{c} \left\{\begin{array}{c} \omega_{jk}^{\prime }=\omega_{jk}+\eta H_{j}\left(L_{k}-Z_{k}\right)\\ \omega_{ij}^{\prime }=\omega_{ij}+\eta H_{j}\left(1-H_{j}\right)x\left(i\right)\overset{m}{\underset{k=1}{\sum }}\omega_{jk}\left(L_{k}-Z_{k}\right) \end{array}\right.\text{.} \end{array}$$

Update the threshold, which is expressed as

(6) $$\begin{array}{c} \left\{\begin{array}{c} \theta_{k}^{\prime }=\theta_{k}+\left(L_{k}-Z_{k}\right)\\ \theta_{j}^{\prime }=\theta_{j}+\eta H_{j}\left(1-H_{j}\right)x\left(i\right)\overset{m}{\underset{k=1}{\sum }}\omega_{jk}\left(L_{k}-Z_{k}\right) \end{array}\right.\text{.} \end{array}$$

### 3.2. Process of BP Neural Network

1. Parameter initialization: set the network structure of the neural network and the number of nodes in each layer, assign random values to the weight matrix and threshold matrix, and assign initial values to parameters such as accuracy and learning rate.
2. Determine the input vector and the target output vector.
3. Calculate the actual output of the hidden layer and the actual output of the output layer.
4. Calculate the error between the target output and the actual output of the output layer. If the error is within the preset range, the learning ends; otherwise, continue with step (5).
5. The weights and thresholds of the hidden layer and the output layer are calculated, respectively.
6. The error signal propagates back along the original direction and modifies the weight and threshold of each layer. Then, it propagates forward from the input layer. The two processes are repeated. If the preset accuracy is reached or the maximum number of learning times is reached, the learning ends. The specific training process is shown in Figure 2.

BP network is the most widely used neural network structure at present, but there are still some problems in the training process:

1. Slow convergence speed: BP algorithm backpropagates the error signal through the network and constantly modifies the weights and thresholds of neurons at each layer until the desired goal is achieved. In other words, the error reduction is at the cost of time.
2. BP algorithm adopts the gradient descent method to adjust the network weight and threshold, so it is easy to fall into the problem of “local minimum.”

## 4. IPSO-BP Neural Network Model

### 4.1. Improved Particle Swarm Optimization (IPSO)

Particle swarm optimization (PSO) is an optimization algorithm based on bird predation. In the optimization calculation, the particle velocity and position are updated by continuously tracking the optimal solution, so as to continuously seek the optimal solution. It is widely used in the solution process of optimization problems [12].

If the particle is regarded as a solution vector in an *N*-dimensional space, assuming that *x* and *v* represent the spatial position and velocity of particle *i*, respectively, the particle update strategy can be expressed as [13]

(7) $$\begin{array}{c} v_{i\;d}\left(t+1\right)=\omega v_{i\;d}\left(t\right)+c_{1}r_{1}\left[p_{id}\left(t\right)-x_{id}\left(t\right)\right]+c_{2}r_{2}\left[p_{gd}\left(t\right)-x_{id}\left(t\right)\right], \end{array}$$

(8) $$\begin{array}{c} x_{id}\left(t+1\right)=x_{id}\left(t\right)+v_{id}\left(t\right), \end{array}$$

where *p*_*id*_(*t*),*p*_*gd*_(*t*) are individual optimal solution and global optimal solution at time *t*; *d* is the dimension of the current particle, *d*=1,2 ⋯ *N*; *ω* is the inertia weight of the particles; *c*_1_,*c*_2_ represent the learning factor; and *r*_1_,*r*_2_ are random numbers evenly distributed between [0, 1].

The traditional particle swarm optimization algorithm is easy to fall into local optimization and exhibits “premature” phenomenon, which affects the addressing accuracy. Therefore, in order to increase the cognitive ability and search range of particles, PSO algorithm is improved. Assuming that variable a is *θ* storage vector, for a particle *i*, select a particle *j* arbitrarily, and the storage vector can be expressed as [14]

(9) $$\begin{array}{c} \theta =p_{id}-x_{j}, \end{array}$$

where *x*_*j*_ is the position of particle *j* at the same time.

Add the storage vector to the addressing process of particles, improve the update strategy of particles, expand the search scope of particles, and solve the problem of “too early maturity.” The update strategy is [15]

(10) $$\begin{array}{c} v_{id}\left(t+1\right)=\left\{\begin{array}{c} \omega \left[v_{id}\left(t\right)+c_{1}r_{1}\theta +c_{2}r_{2}\left(p_{gd}\left(t\right)-x_{id}\left(t\right)\right)\right]\\ \omega \left[v_{id}\left(t\right)+c_{1}r_{1}\left(p_{id}\left(t\right)-x_{id}\left(t\right)\right)+c_{2}r_{2}\left(p_{gd}\left(t\right)-x_{id}\left(t\right)\right)\right] \end{array}\right.\text{.} \end{array}$$

### 4.2. Training Process of IPSO-BP Neural Network

As an optimization tool, PSO is an optimization algorithm based on swarm intelligence theory. Combining PSO with neural network, PSO algorithm is used to optimize the weight and threshold of neural network, and the swarm intelligence generated by particle cooperation and competition is used to guide the optimization search, so as to improve the performance of BP algorithm. The optimized algorithm has fast convergence speed, good robustness, and strong global search ability. Moreover, the addressing process no longer depends on gradient information, avoids the requirements of gradient descent method on function, shortens the training time of neural network, and greatly improves the search efficiency.

The fusion of IPSO algorithm and BP algorithm is mainly reflected in two aspects. Firstly, the position vector of particles in IPSO algorithm will correspond to all connection weights and thresholds of BP algorithm and find the optimal position through fitness function, that is, find the optimal weight and threshold of BP network. Secondly, the forward propagation theory of BP neural network is used to calculate the particle fitness, and the particle fitness function is defined according to the trained mean square error [16]. The training steps of IPSO-BP neural network are as follows:

1. By analyzing the sample data, the BP network model is constructed.
2. Input training data to determine the fitness function value of each particle.
3. Parameter initialization: assign values to each parameter.
4. Update the velocity and position of the particle swarm according to formulas (7)–(10).
5. Iterative operation: if the current fitness value is better than the local optimal value of particle swarm optimization, it will be replaced to update the local optimal solution of particle swarm optimization.
6. The global optimal position vector is mapped to the weight and threshold of BP neural network.
7. Input the samples to be predicted into the optimized network model and analyze the prediction results.

The specific process is shown in Figure 3.

### 4.3. Training Results and Analysis

In order to verify the scientificity of the teaching quality evaluation index system and the reliability of IPSO-BP model, 2000 pairs of input and output data are randomly generated by the program between [0,1] on the MATLAB platform as training samples, and the data are trained by BP neural network and IPSO-BP neural network, respectively.

This paper adopts a three-layer BP neural network framework. There are 16 nodes in the output layer, 5 nodes in the hidden layer, and 1 node in the output layer.

In the process of setting model parameters, the calculation formula of particle dimension is

(11) $$\begin{array}{c} D=I\times H+H\times O+H+O\text{,} \end{array}$$

where *I* is the number of neurons in the input layer; *H* is the number of neurons in the hidden layer; and *O* is the number of neurons in the output layer.

Calculate the particle dimension according to formula (11), D = 16) × 5 + 5 × 1 + 5 + 1 = 11. Because the number of particles has a great impact on the final optimization results, if it is too small, the search range is limited, the optimization accuracy is low, and the “premature” problem is easy to occur. If it is too large, the algorithm is complex, which will greatly reduce the optimization efficiency. Therefore, in this paper, the number of particles is taken as *N* = 60. The maximum number of iterations is 500. The learning factor is as follows: *C*_1_ = 1.5, *C*_2_ = 2. The maximum and minimum values of inertia weight are 0.8 and 0.3, respectively. The speed range is [−1, 1]. The transfer function of neurons in hidden layer and output layer is sigmoid function, and Traingd function is used for network training. The target error of the network is 0.001. When the training error is less than the target error, the training ends. The results are shown in Figures 4 and 5.

Mean square error (MSE), prediction accuracy, training time, and iteration times are used as evaluation performance indicators for analysis and compared with the BP model. The results are shown in Table 2.

It can be seen that compared with BP neural network model, the IPSO-BP model has fast convergence speed and can find the optimal solution in less iterations. At the same time, the training error of the model is small, and a better prediction accuracy can be obtained. The training results show that the IPSO-BP neural network model has certain reliability and effectiveness and can be used to evaluate the quality of classroom teaching.

## 5. Teaching Quality Evaluation Based on IPSO-BP Neural Network Model

### 5.1. Evaluation Grade Division

According to the expert experience and the actual situation of the course teaching effect, the evaluation results are divided into five levels, namely, “excellent, good, medium, pass, and fail,” and the value range of each level is specified, as shown in Table 3.

### 5.2. Collection of Sample Data

In order to construct the sample data needed in the training process of IPSO-BP neural network model, six professional courses of animal science major of Inner Mongolia University for Nationalities from 2020 to 2021 are selected as the object of teaching quality evaluation, the comprehensive score of the attendance results of school supervisors is taken as the expected output, and the questionnaire score results of students in class are taken as the training data. In order to reduce the demand of the network for samples, firstly, the training results need to be normalized to keep the results between [0, 1]. The normalization calculation formula is

(12) $$\begin{array}{c} z=\frac{x-\min\left(x_{i}\right)}{\max\left(x_{i}\right)-\min\left(x_{i}\right)}\text{.} \end{array}$$

First of all, experts are invited to evaluate the listening results of six professional courses: 《Animal anatomy》, 《Animal physiology》, 《Animal nutrition》, 《Animal genetics》, 《Animal reproduction》, and 《Feed science》. Secondly, a questionnaire is distributed to students to examine the teaching effect of each course, so as to obtain sample data. Then, the IPSO-BP neural network model is trained by using the sample data of the first five courses, and the model is optimized according to the expert evaluation results. Finally, the trained model is used to test and evaluate the last course to test the effectiveness of the evaluation model. A total of 222 valid samples were received in the questionnaire. The first 192 samples were used for the training of IPSO-BP neural network model, and the last 30 results were used for the test of network generalization ability. The evaluation results of experts in each course and the number of questionnaires are shown in Table 4.

### 5.3. Evaluation Results and Analysis

Input 192 sample data of the first five courses into IPSO-BP network model for training and complete the training after approaching the evaluation index. The training results of some samples are shown in Table 5.

In Table 5, taking the teaching quality evaluation results of《Animal anatomy》course as an example, among the evaluation indicators, “innovative ability training (*A*_32_)” has the best evaluation results, and the indicator “teaching ideas (*A*_22_)” has poor evaluation results and needs to be improved in this regard, but the overall evaluation grade is “excellent.”

In order to further discuss the effectiveness of IPSO-BP neural network model, the modeling time and evaluation accuracy in the evaluation process are graphically represented and compared with BP neural network and PSO-BP neural network, as shown in Figures 6 and 7.

The results show that compared with the other two models, the IPSO-BP neural network model has fast modeling speed and can greatly reduce the network running time. At the same time, the accuracy rate of the teaching quality evaluation of the model is more than 94%, while the accuracy rate of the BP model is the least, less than 85%. It shows that IPSO algorithm can not only solve the “premature” phenomenon of PSO algorithm but also effectively optimize the weight and threshold of neural network, so as to improve the performance of BP algorithm and meet the application requirements of teaching quality evaluation.

### 5.4. Testing and Verification

The purpose of model training is application, so it is necessary to test the trained model to verify the generalization ability of the trained network model. 30 data samples of “Feed science” course are tested in the trained IPSO-BP neural network model and compared with the BP neural network model. The test results of some samples are shown in Table 6.

In order to analyze the test results more intuitively, the results in Table 6 are represented by curves, as shown in Figures 8 and 9.

It can be seen that among all 30 test samples, the IPSO-BP neural network model has 29 samples with correct judgment, only one sample has wrong judgment, and the evaluation accuracy is 96.7%, while BP neural network model has 4 samples with wrong judgment, and the evaluation accuracy is 86.7%. The test results show that the IPSO-BP neural network model constructed in this paper can greatly improve the prediction accuracy and has strong generalization ability. It can obtain better evaluation results when it is used in the evaluation of teaching quality.

## 6. Conclusions

1. Aiming at the problems of BP neural network, an IPSO-BP neural network model is constructed. The improved particle swarm optimization algorithm is used to optimize the weight and threshold of neural network, so as to improve the performance of BP algorithm. The simulation results show that the model has the advantages of fast operation speed and high addressing accuracy.
2. Taking teaching attitude, teaching content, teaching method, and teaching effect as indicators, the teaching quality evaluation index system is established. Taking the animal science major of Inner Mongolia University for Nationalities as an example, the sample set is constructed, and the IPSO-BP neural network model is used for sample training and testing.
3. The results show that compared with other models, the IPSO-BP neural network model has fast convergence speed, good robustness, 96.7% prediction accuracy, and strong generalization ability. At the same time, it further verifies the effectiveness of the established evaluation index system and provides a new way for teaching quality evaluation.

## Figures and Tables

**Figure 1:** Basic structure of BP neural network.

**Figure 2:** Training process of BP neural network.

**Figure 3:** IPSO-BP neural network training process.

**Figure 4:** Running time of different models.

**Figure 5:** MSE of different models.

**Figure 6:** Modeling time comparison.

**Figure 7:** Accuracy comparison.

**Figure 8:** Prediction results of BP neural network model.

**Figure 9:** Prediction results of IPSO-BP neural network model.

**Table 1:** Teaching quality evaluation index system.

Primary index	Weight	Secondary index	Weight
Teaching attitude (A1)	0.21	Mental outlook (A11)	0.18
		Preparation before class (A12)	0.34
		Attendance rate (A13)	0.27
		Professionalism (A14)	0.21

Teaching contents (A2)	0.23	Teaching objectives (A21)	0.21
		Teaching ideas (A22)	0.32
		Key points and difficulties (A23)	0.22
		Logic and clarity (A24)	0.25

Teaching method (A3)	0.27	Diversification of teaching methods (A31)	0.26
		Cultivation of innovation ability (A32)	0.28
		Students as the main body (A33)	0.24
		Combining theory with practice (A34)	0.22

Teaching effectiveness (A4)	0.29	Classroom atmosphere (A41)	0.21
		Teacher student interaction (A42)	0.19
		Knowledge mastery (A43)	0.32
		Problem solving ability (A44)	0.28

**Table 2:** Comparison of training results.

Model	Running time (s)	Accuracy (%)	MSE	Number of iterations
BP model	24.08	85.8	0.0927	364
IPSO-BP model	8.95	96.2	0.0613	243

**Table 3:** Evaluation grade division.

Grade	Excellent	Good	Medium	Pass	Fail
Value range	0.90∼1.00	0.80∼0.89	0.70∼0.79	0.60∼0.69	0∼0.59

**Table 4:** Evaluation results of experts in each course and the number of questionnaires.

Course name	Number of questionnaires	Expert evaluation results	Expert evaluation score
《Animal anatomy》	35	Excellent	0.93
《Animal physiology》	38	Good	0.86
《Animal nutrition》	43	Medium	0.77
《Animal genetics》	40	Good	0.84
《Animal reproduction》	36	Excellent	0.94
《Feed science》	30	Good	0.87

**Table 5:** Training results of some samples.

Course name	Sample number	Actual output	Expected output	Training results	Expert results
《Animal anatomy》	1	0.9523	0.95	Excellent	Excellent
	2	0.9486	0.95	Excellent	Excellent
	…				
	35	0.9535	0.95	Excellent	Excellent

《Animal physiology》	1	0.8482	0.85	Good	Good
	2	0.8627	0.85	Good	Good
	…				
	38	0.8545	0.85	Good	Good

《Animal nutrition》	1	0.776	0.75	Medium	Medium
	2	0.7486	0.75	Medium	Medium
	…				
	43	0.7683	0.75	Medium	Medium

《Animal genetics》	1	0.8369	0.85	Good	Good
	2	0.8454	0.85	Good	Good
				
	40	0.8531	0.85	Good	Good

《Animal reproduction》	1	0.9317	0.95	Excellent	Excellent
	2	0.9532	0.95	Excellent	Excellent
	…				
	36	0.9478	0.95	Excellent	Excellent

**Table 6:** Test sample of partial sample.

Course name	Sample number	BP output result	IPSO-BP output results	Expected output
《Feed science》	1	0.8258	0.8376	0.84
	**2**	0.9235	0.9001	0.88
	3	0.8316	0.8316	0.84
	4	0.8428	0.8428	0.85
	5	0.7932	0.8376	0.83
	6	0.8968	0.8771	0.88
		… … …		
	30	0.8737	0.8528	0.85

## Data Availability

The data used to support the findings of this study are available from the corresponding author upon request.
